The article "Imaging Features and Pathological Analysis of 43 Parotid Basal Cell Adenomas" was published in 2021. Journal: Comput Math Methods Med.

# Imaging Features and Pathological Analysis of 43 Parotid Basal Cell Adenomas

**DOI:** 10.1155/2021/7906058

**Published:** 2021-12-06

**Authors:** Guiqin Chen, Xiaoyi Wen, X. J. Chen, Lei Zhang, Z. T. Lin, Lei Jing, Tiemei Wang

**Affiliations:** ^1^Department of Ultrasound, Nanjing Stomatological Hospital, Medical School of Nanjing University, Nanjing, China; ^2^Department of Pharmacy, Children's Hospital of Nanjing Medical University, Nanjing, China; ^3^Department of Dentomaxillofacial Pathology, Nanjing Stomatological Hospital, Medical School of Nanjing University, Nanjing, China; ^4^Department of Dentomaxillofacial Radiology, Nanjing Stomatological Hospital, Medical School of Nanjing University, Nanjing, China; ^5^Department of Ultrasound, The First Affiliated Hospital of Nanjing Medical University, Nanjing, China

## Abstract

**Purpose:**

To investigate the correlation between sonographic and computed tomography and pathological features of basal cell adenomas (BCAs) of the parotid gland.

**Methods:**

This retrospective study included 41 patients (43 tumors) with BCAs. The tumors were divided into three types based on their location in the parotid gland and their imaging features. The features of the tumors were analyzed.

**Results:**

Imaging manifestations and corresponding pathological results of most BCAs of the parotid glands resembled those of benign parotid gland tumors. Malignant transformation occurred in membranous BCAs and in those with extensive cribriform structures. Type-II and type-III tumors accounted for 82.93% of the total proportion. Thirteen tumors showed cystic degeneration with 30.23%, among which type-III tumors could easily develop cystic degeneration. These cystic areas might correspond to cystic degeneration or focal necrosis. Cystic change was not dependent on the tumor size. The pathological features of the tumors were correlated to their imaging manifestations.

**Conclusion:**

Most BCAs of the parotid glands have imaging manifestations similar to those of benign parotid gland tumors. BCAs with extensive cribriform structures and of the membranous type can show malignant transformation and should be treated with caution in clinical practice.

## 1. Introduction

Parotid tumors account for approximately 3% of all head and neck neoplasms. Basal cell adenoma (BCA) of the salivary gland is a rare benign epithelial tumor that most frequently occurs in the parotid gland and ranks third among benign parotid tumors [1, 2]. BCA was described as a new distinct histological entity by the World Health Organization in 1991 and classified as one of nine salivary gland cancers in 2005 [3] and has been extensively researched since then. BCA is composed of monomorphic basaloid cells without a myxochondroid component and is classified into four subtypes according to cell arrangement, i.e., solid, trabecular, tubular, and membranous. Membranous BCAs are relatively rare and are considered malignant with a high recurrence rate at approximately 24% and more common malignant transformation, even if extremely rare at 4.3%, whereas the other types are considered benign with nearly zero rates of recurrence and malignant transformation [4]. In our experience, the imaging features of most basal cell tumors resemble those of other benign tumors of the parotid glands and of the three types (i.e., solid, trabecular, and tubular) in pathology. However, we have encountered several cases that acted as malignant tumors, and the pathology showed potential malignancy, two of the three types (i.e., solid, trabecular, and tubular) and one of the membranous type. Therefore, the imaging and pathological features of such BCAs merit investigation. In the present study, we examined the disease course, clinical manifestations, tumor treatment, sonographic, computed tomography (CT), and pathological features, and follow-up results of 43 parotid BCAs in 41 patients.

## 2. Materials and Methods

This retrospective study included 41 patients with parotid BCAs who underwent surgery in our hospital between September 2017 and August 2019. Approval for this study was received from the institutional review board, and the requirement for informed consent was waived due to the retrospective nature of the study.

All patients with parotid-gland tumors as the chief complaint were admitted to our hospital and underwent preoperative sonography (ALOCKA *α*7, Tokyo, Japan, and Esaote MyLab ClassC, Genova, Italy) and CT (Siemens Definition AS, Erlangen, Germany) scanning; biopsy was not performed before the sonography and CT scanning in any case. Partial or complete parotidectomy followed these examinations according to the pathology. Tumors were examined by routine pathology and immunohistochemistry [5]. We reviewed, collected, and analyzed all data, including sex, age, symptoms, sonography, CT, surgical details, pathology, and immunohistochemistry. Hematoxylin and eosin staining was used to determine the arrangement of basaloid epithelial cells, which revealed a distinctive basement membrane-like material, and immunohistochemistry was used to examine the presence of epithelial membrane antigen, transformation-related protein 63, soluble protein-100, ck 5/6, ck 8/18, CD117, calponin, and Ki-67.

According to their location in the parotid gland, the tumors were divided into three types as follows: type I and type II located in the superficial lobe of the parotid gland and type III located in the deep lobe of the parotid gland. The superficial and deep lobes of the parotid gland were separated by the retromandibular vein. The superficial lobe was further divided into two types, namely, type I, close to the superficial border of the superficial lobe, and type II, close to the retromandibular vein in the superficial lobe.

### 2.1. Statistical Analysis

Statistical analysis was performed using SPSS statistical software v. 17.0 (SPSS Inc., Chicago, IL) using the chi-squared test. A *P* value < 0.05 was considered statistically significant.

## 3. Results

As shown in Table 1, of the 41 included patients, 26 (63.41%) were women and 15 (36.59%) were men with an average age of 57.67 ± 3.56 years (range, 20–86 years); the percentage of patients aged >55 years was 58.54%, whereas that of those aged >60 years was 36.59%. The tumors were located on the left side in 14 patients and on the right side in 27 patients. There were no significant differences in sex, age, or side for all types of tumors (chi-squared test, *P* > 0.05). There were seven type-I, 12 type-II, and 24 type-III masses. The smallest mass was a type I sized 0.8 × 0.7 cm, and the largest mass was a type III sized 4.7 × 2.8 cm. The mean size to diameter of type-I tumors was 1.21 ± 0.64 cm, that of type-II tumors was 2.14 ± 1.08 cm, and that of type-III tumors was 2.33 ± 2.72 cm. According to the pathology, there were 11 solid, 1 membranous, 13 tubular, 10 trabecular, 5 solid–tubular, and 3 solid–trabecular masses. Two patients had multiple nodules on one side of the parotid gland. The shape of most masses was regular, e.g., ovoid; however, two type-III tumors extended from the deep lobe of the parotid gland to the upper part of the neck. The oblong diameter of the biggest tumor was 4.7 cm, and its capsule showed eggshell-like calcification; it was closely related to the carotid artery. The mean disease duration of type-I tumors was 17.6 ± 2.2 months, that of type-II tumors was 21 ± 3.9 months, and that of type-III tumors was 20 ± 5.1 months. The capsules of 40 tumors were clear. There were 13 masses with cystic changes, of which 8 were type III (in the deep lobe), 3 were type II, and 2 were type I. Type-III tumors were more likely to have cystic changes (8/24, 33.33%) than type-II (3/12, 25%) and type-I (2/7, 28.57%) tumors. Most tumors showed clear boundaries and regular shapes; 30 masses were hypoechoic, of which, 26 were homogeneous, and 13 of the total 43 masses showed mixed echogenicity, including hypoechoic and cystic changes. Forty tumors showed posterior echo enhancement, similar to the imaging features of benign parotid tumors. Twenty-six masses were hypervascular, whereas 17 masses were not. Plain CT scanning showed mostly regular masses with uniform density.

During the clinical examination, we also found that three masses were ill-defined and heterogeneous or showed calcification and hypervascularization. Determination of malignancy was easy due to the ill-defined borders, heterogeneity, and hypervascularization. In plain CT, these three masses were found to be of regular shape with unclear boundaries, low density, and heterogeneity. To identify them, we carefully examined the hematoxylin and eosin staining and immunohistochemical results of the three masses and found one case of membranous-type BCA (Figure 1), one of the trabecular type with extensive cribriform structures (Figure 2), and one solid with extensive cribriform structures (Figure 3). The membranous-type BCA invaded the capsule. The trabecular mass with extensive cribriform structures invaded the nerves, and the solid mass with extensive cribriform structures invaded the fat cells in the surrounding tissue. Complete parotidectomy was performed, followed by close clinical observation, as is the standard in such cases, which tend to be multicentric, have multiple recurrences, and occasionally undergo malignant transformation [6]. All patients were followed up at 3 and 6 months postoperatively, and no local recurrence, malignant transformation, or distant metastasis was found. In addition, we found two multinodular cases, which is very rare.

Immunohistochemical examination showed positive results for soluble protein-100, transformation-related protein 63, ck 5/6, ck 8/18, CD117, and calponin (Figure 4) in all cases, which were some epithelial membrane antigens. The value of Ki-67, a marker of cell proliferation, was <5%.

## 4. Discussion

BCAs are rare benign tumors that mostly appear in the parotid glands of elderly women [1, 4, 5]. The proportion of younger patients with BCAs was higher in this study than in previous studies that reported that BCA is more often found in women aged >60 years [2, 7]. In addition, in this study, most tumors were located on the right side of the gland, whereas previous studies have reported greater frequency of tumors located on the left side [8, 9]. Two patients had multiple nodules in the left parotid gland. Although BCA and oncocytoma may also be multifocal and unilateral, Warthin's tumor is the most common multifocal unilateral neoplasm [10]. Therefore, the two types should be carefully distinguished.

The shape of most tumors of all types in this study was regular. Some type-III BCAs could be easily confused with a carotid body tumor and should, therefore, be distinguished in combined assessment with other clinical findings and imaging features. For example, carotid body tumors have pulsations; computed tomography angiography could be sometimes used to distinguish between the tumor types. It appears that the average size of the three types of tumors reported herein increased in order, which is consistent with previously reported findings [11].

In this study, type-II and type-III tumors accounted for 82.93% of the total proportion, indicating that BCAs occur in the deep superficial lobe or deep lobe of the parotid gland. Thirteen tumors showed cystic degeneration, i.e., two, three, and eight of type-I, type-II, and type-III tumors, respectively, suggesting that type-III tumors could easily develop cystic degeneration. The ratio of cystic degeneration in this study was 30.23%, which was similar to that reported in previous studies [1, 12]. Most previous studies have reported that cystic areas are more frequently present in Warthin's tumors than in pleomorphic adenomas. Some studies have noted a high frequency of anechoic areas in Warthin's tumors, at 44.8–93.3% [13, 14]. These cystic areas might correspond to cystic degeneration or focal necrosis [15]. Cystic changes originating from hemorrhage are often noted in larger pleomorphic adenomas [16], and the same mechanisms may be implicated in focal necrosis or hemorrhage seen in BCAs and cystic degeneration.

Immunohistochemical examination showed positive results for soluble protein-100, transformation-related protein 63, ck 5/6, ck 8/18, CD117, and calponin (Figure 4) in all cases, which were some epithelial membrane antigens. The value of Ki-67, a marker of cell proliferation, was <5%.

In this study, cystic change was not dependent on the tumor size; for instance, the largest observed tumor showed no cystic change, which is in agreement with the findings of previous reports. We found that 40 tumors showed distal acoustic enhancement, whereas 3 did not. Kovacevic and Fabijanic reported that the ultrasonographic feature that is most often associated with benign lesions is distal acoustic enhancement [11], which is shown by most parotid benign tumors. Most of the tumors (*n* = 40) in our study showed clear boundaries and capsule, regular shape, and uniform anechoic or hypoechoic echoes or hypoechogenicity with cystic changes, enhanced posterior echo, and abundant flow on color Doppler flow imaging, similar to the imaging manifestations of benign parotid tumors. In this study, plain CT showed regular masses with uniform or uneven density. Moreover, we found early intense BCA enhancement for most masses with CT enhancement; in the venous phase, some masses continued to appear enhanced, whereas some did not. This phenomenon might be related to the tumor's vascular architecture. The solid component of BCAs includes numerous endothelium-lined vascular channels, with prominent small capillaries and venules [17].

During clinical examination, we also found three masses with ill-defined borders, heterogeneous echo, and calcification with rich blood flow, which were easily diagnosed as malignant due to the poorly defined borders, heterogeneity, and mixed echotexture [18, 19]. Spot-like or needlelike calcification can be caused by local abnormal calcium and phosphorus metabolism in malignant tumors or by long-standing pleomorphic adenomas [20]. Well-vascularized masses mostly indicate malignant tumors. The most common malignant tumors are mucoepidermoid carcinoma and adenoid cystic carcinoma, followed by adenocarcinoma, squamous cell carcinoma, and lymphoma [21, 22]. All these malignant tumors, except lymphoma, are mainly composed of epidermoid and basal-like cells; facial nerve paralysis and metastatic lymph nodes are commonly associated with such tumors but were not observed in any of the abovementioned three masses in this study. Malignant transformation is more common in the membranous type, appearing in approximately 4.3% of cases [4]. The membranous type is multifocal, with a multinodular growth pattern, and recurrences are common (24%) [23]. BCAs with extensive cribriform structures may have potential of low-grade malignancy and extend to the capsule or surrounding tissues even when they are not of the membranous types. Moreover, BCAs with extensive cribriform structures may have imaging features similar to those of malignant tumors and act in a manner resembling the membrane types invading the surrounding tissues.

This study had several limitations. First, it was retrospective and, thus, ultrasonographic features were not evaluated in real-time. Second, the sample size was small, with only 43 tumors; therefore, further larger studies are required. Third, we relied on the accuracy of the pathological diagnosis and excluded patients who had not undergone surgery. However, the images were interpreted together by two investigators, preventing the assessment of interobserver variability.

In conclusion, BCA of the parotid gland tends to appear in elderly women, is located in the deep lobe of the parotid gland, and often involves cystic changes. The imaging manifestations and corresponding pathological results of most BCAs of the parotid glands resemble those of benign parotid gland tumors. Further, BCAs with extensive cribriform structures and of the membranous type could show malignant transformation, which should be treated with caution in clinical practice. Thus, if a mass with cystic degeneration is detected in the deep lobe of the parotid gland, the possibility of it being a BCA should be considered.

## Figures and Tables

**Figure 1:** A 20-year-old woman with a membrane-type BCA. (a) Transverse grayscale ultrasonographic image of a 20-year-old woman. There is an ill-defined, regular, hypoechoic mass with heterogeneous internal architecture and without posterior enhancement in the right parotid gland. (b) Intramodular prominent vascularity on Doppler B. (c) Plain computed tomography scan showing an ill-defined regular mass with uneven low density. (d) Hematoxylin and eosin (HE) staining: (membrane type) thickened basement membrane-like substance around a cell mass (×200), scar bar. (e) HE staining: tumor cells invade the capsule (×100).

**Figure 2:** A 68-year-old woman with a trabecular-type BCA. (a) A 68-year-old woman with a regular, ill-defined, hypoechoic, heterogeneous mass without posterior enhancement in the right parotid gland. (b) Intramodular prominent vascularity on Doppler B. (c) Plain computed tomography scan showing a regular, ill-defined mass with uneven low density. One of the trabecular type with extensive cribriform structures. (d) Computed tomography angiography (CTA): continuous heterogeneous enhancement in the arterial and venous phases. (e) (trabecular) neoplastic basal-like cells are arranged in a cord-like structure (×200). (f) Trabecular mass with extensive cribriform structures (×200); Scar bar. (g) Tumor cells invading the nerves (×100).

**Figure 3:** A 56-year-old woman of a solid-type BCA. (a, b) Transverse grayscale ultrasonographic image of a 56-year-old woman. An ill-defined, regular, mixed echo mass with heterogeneous internal architecture and with calcification without light posterior enhancement in the right parotid gland. (c) A small amount of blood on Doppler B. (d) Plain computed tomography scan showing a regular, ill-defined, uneven mass with low density and calcification. (e, f) (solid) Tumor cells are arranged in a sheet or island structure, and some are with heteromorphic; extensive cribriform structures are present (×200); Scar bar. (g) Tumors are invading the fat cells (×100).

**Figure 4:** Immunohistochemistry of BCA: (a) CD 117 (×200); (b) ck 5/6 (×200); (c) ck 8/18 (×200); (d) transformation-related protein 63 (×200); (e) soluble protein-100 (×200); (f) calponin (×200). Scar bar.

**Table 1:** Patient and tumor characteristics by type.

	Tumor	Sex	Age	Side	Disease duration	Size (cm)	Shape	Margin	Echogenicity	Echotexture	Cystic formation	Enhanced Posterior echo	Vascularized	Pathology	
Type I	7	Female = 4 Male = 3	56.57 ± 4.01	L = 3 R = 4	17.6 ± 2.2	1.21 ± 0.64	Ovoid = 7 Lobulated = 0	Well‐defined = 7 Ill‐defined = 0	Hypoechoic = 5 Mixed = 2	Homogeneous = 4 Heterogeneous = 3	2 (28.57%)	Present = 7 Absent = 0	Hypovascular = 4 Hypervascular = 3	Solid = 2 Tubular = 3 Trabecular = 1 Membrane = 0 Solid tubular = 1	
Type II	12	Female = 6 Male = 6	51.92 ± 3.12	L = 3 R = 9	21.00 ± 3.9	2.14 ± 1.08	Ovoid = 10 Lobulated = 2	Well‐defined = 11 Ill‐defined = 1	Hypoechoic = 9 Mixed = 3	Homogeneous = 7 Heterogeneous = 4 Calcification = 1	3 (25%)	Present = 10 Absent = 2	Hypovascular = 4 Hypervascular = 8	Solid = 3 Tubular = 2 Trabecular = 3 Membrane = 1 Solid tubular = 2 Solid trabecular = 1	
Type III	24	Female = 16 Male = 6	57.73 ± 3.89	L = 8 R = 14	20.00 ± 5.1	2.33 ± 2.72	Ovoid = 24 Lobulated = 0	Well‐defined = 22 Ill‐defined = 2	Hypoechoic = 16 Mixed = 8	Homogeneous = 15 Heterogeneous = 8 Calcification = 1	8 (33.33%)	Present = 23 Absent = 1	Hypovascular = 9 Hypervascular = 15	Solid = 6 Tubular = 8 Trabecular = 6 Membrane = 0 Solid tubular = 2 Solid trabecular = 2	
Total	43	Female = 26 (63.41%) Male = 15 (36.59%)	57.67 ± 3.56	L = 14 (34.15%) R = 27 (65.85%)	18.52 ± 4.5	2.13 ± 1.28	Ovoid = 41 Lobulated = 2	Well‐defined = 40 Ill‐defined = 3	Hypoechoic = 30 Mixed = 13	Homogeneous = 26 Heterogeneous = 15 Calcification = 2	13 (30.23%)	Present = 40 Absent = 3	Hypovascular = 17 (39.53%) Hypervascular = 26 (60.47%)	Solid = 11 Tubular = 13 Trabecular = 10 Membrane = 1 Solid tubular = 5 Solid trabecular = 3	
	/	/	*P* > 0.05	/	*P* > 0.05	*P* > 0.05	/	/	/	/	/	/	/	/	

L: left; R: right.

## Data Availability

The data used during the present study are available from the corresponding author upon reasonable request.
